This article has been retracted.

# Age Related Changes in NAD+ Metabolism Oxidative Stress and Sirt1 Activity in Wistar Rats

**DOI:** 10.1371/journal.pone.0019194

**Published:** 2011-04-26

**Authors:** Nady Braidy, Gilles J. Guillemin, Hussein Mansour, Tailoi Chan-Ling, Anne Poljak, Ross Grant

**Affiliations:** 1 Department of Pharmacology, School of Medical Sciences, Faculty of Medicine, University of New South Wales, Sydney, Australia; 2 St Vincent's Centre for Applied Medical Research, Sydney, Australia; 3 Retinal and Developmental Neurobiology Lab, Discipline of Anatomy and Histology, School of Medical Sciences, University of Sydney, Australia; 4 Bioanalytical Mass Spectrometry Facility, University of New South Wales, Sydney, Australia; 5 Australasian Research Institute, Sydney Adventist Hospital, Sydney, Australia; University of Hong Kong, China

## Abstract

The cofactor nicotinamide adenine dinucleotide (NAD+) has emerged as a key regulator of metabolism, stress resistance and longevity. Apart from its role as an important redox carrier, NAD+ also serves as the sole substrate for NAD-dependent enzymes, including poly(ADP-ribose) polymerase (PARP), an important DNA nick sensor, and NAD-dependent histone deacetylases, Sirtuins which play an important role in a wide variety of processes, including senescence, apoptosis, differentiation, and aging. We examined the effect of aging on intracellular NAD+ metabolism in the whole heart, lung, liver and kidney of female wistar rats. Our results are the first to show a significant decline in intracellular NAD+ levels and NAD∶NADH ratio in all organs by middle age (i.e.12 months) compared to young (i.e. 3 month old) rats. These changes in [NAD(H)] occurred in parallel with an increase in lipid peroxidation and protein carbonyls (o- and m- tyrosine) formation and decline in total antioxidant capacity in these organs. An age dependent increase in DNA damage (phosphorylated H2AX) was also observed in these same organs. Decreased Sirt1 activity and increased acetylated p53 were observed in organ tissues in parallel with the drop in NAD+ and moderate over-expression of Sirt1 protein. Reduced mitochondrial activity of complex I–IV was also observed in aging animals, impacting both redox status and ATP production. The strong positive correlation observed between DNA damage associated NAD+ depletion and Sirt1 activity suggests that adequate NAD+ concentrations may be an important longevity assurance factor.

## Introduction

Multiple degenerative processes are implicated in natural senescence. As aging is associated with progressive decline in organ function, elucidating the complex pathways controlling the rate of aging is of significant clinical importance [1]. An important mechanism contributing to aging is oxidative stress. The “free-radical theory of aging”, initially proposed by Harman (1956) suggests that oxidative damage occurs with advanced aging due to an imbalance between free radical and reactive species (ROS) production, and cellular antioxidant defense mechanisms [2]. Elevated levels of intracellular ROS through hydrogen peroxide treatment, or deficiency of ROS scavenging enzymes such as superoxide dismutase (SOD1) knockdown, has been shown to induce premature senescence and reduce cellular life span [3], [4], [5].

The mitochondria, represents the main producer of cellular ROS in the human body, and approximately 1–2% of the oxygen molecules consumed during normal respiration are converted into highly reactive superoxide anion, which is rapidly dismutated to H_2_O_2_ by the superoxide dismutases [6]. Other pathways and events able to produce ROS include peroxisomal metabolism, enzymatic synthesis of nitric oxide, phagocytic leukocytes, heat, ultraviolet (UV) light, therapeutic drugs, and ionizing radiation [7]. Intracellular ROS, due to their high reactivity, can interact with a spectrum of biological molecules, leading to the oxidation of several macromolecules, such as protein, lipids, and nucleic acids [8]. As a result, vital functions, such as energy production, maintenance of plasma membrane potential, and cellular ionic homeostasis may be impaired in the early stage of oxidative stress [8]. Excessive oxidative insult may also stimulate secondary events leading to cell death via an apoptotic mechanism [9].

A major factor associated with age-related diseases is the increase of oxidative DNA damage [7]. It is estimated that at least 5000 single-stranded DNA breaks occur during a single cell cycle as a result of ROS production [10], [11]. Approximately 1% of these DNA breaks are converted into double-stranded DNA breaks, primarily during DNA replication. Accumulation of unrepaired DNA damage induced by ROS can lead to arrest or induction of transcription, induction of signal transduction pathways, replication errors and genomic instability [10], [11]. These molecular changes are observed in both cancer and aging, and this supports the notion that chronic oxidative damage to DNA might trigger cancer and promote aging [10], [11].

The removal of oxidative DNA damage through repair of DNA single strand breaks by DNA base excision repair, is facilitated by Poly(ADP-ribose) polymerase-1 (PARP) [12], [13], [14]. PARP is an abundant protein modifying nuclear enzyme involved in DNA repair. The enzymatic activity of PARP is strongly activated in cells in response to treatment with ROS such as H_2_O_2_ [15]. Activation of PARP leads to the transfer of ADP-ribose moieties from NAD^+^, to the target protein [16]. Since PARP uses NAD^+^ as the only endogenous substrate for poly-ADP-ribosylation, PARP activity is dependent on the amount of NAD^+^ available, and may act as a nuclear energy sensor. Under physiological conditions, mild activation of PARP can regulate several cellular processes, including DNA repair, cell cycle progression, cell survival, chromatin remodeling, and genomic stability [13], [17]. However, overactivation of PARP can repress genomic transcription and reduce cell survival. NAD^+^, in addition to being a substrate for PARP, also serves as an important redox carrier to power oxidative phosphorylation and ATP production [18]. Depletion of NAD^+^ following PARP hyperactivation has been shown to deplete intracellular ATP stores leading to the release of apoptosis-inducing factors (AIF) and consequent cell death due to energy restriction [19]. PARP activation has been implicated in the pathogenesis of hypertension, atherosclerosis, lung injury, haemorrhagic shock, and diabetic cardiovascular and kidney complications [20], [21], [22], [23], [24]. In these diseases, the oxidant-mediated endothelial cell injury is dependent on PARP activation, and can be attenuated by pharmacological PARP inhibitors [25], [26]. Therefore, tight regulation of PARP activity is crucial to prevent the development of several age-related pathological disorders.

In addition to its role in PARP activity, another essential factor that is greatly affected by changes in intracellular NAD^+^ levels is the class III histone deacetylases known as sirtuins, or silent information regulator of gene transcription [27]. Gene silencing by this family of enzymes has been correlated directly with longer lifespan in yeast and worms [28]. In yeast, sir2 plays a critical role in transcriptional silencing and maintenance of genomic stability [29], [30]. Sirt1 is the human homolog of sir2 and appears to be involved in several physiological functions including the control of gene expression, cell cycle regulation, apoptosis, DNA repair, metabolism, and aging [31], [32], [33]. Sirt1 can deacetylate numerous proteins such as tumor suppressor protein, p53, which modulates various genes that control damaged DNA [34]. The deacetylase activity of SIRT proteins is dependent on the intracellular NAD^+^ content [27]. They catalyse a unique reaction that releases nicotinamide, acetyl ADP-ribose (AADPR), and the deacetylated substrate [27]. Impaired SIRT1 activity due to PARP mediated NAD^+^ depletion allows increased activity of several apoptotic effectors such as p53, therefore sensitising cells to apoptosis. Adequate NAD^+^ levels are therefore critical to maintaining Sirt1 activity which can delay apoptosis and provide vulnerable cells with additional time to repair even after repeated exposure to oxidative stress [35].

Though a number of studies have demonstrated elevated levels of oxidative stress associated damage in aged tissue, to our knowledge, no study has yet reported on changes in NAD^+^ levels during the aging process. In this study, we have characterized and quantified changes in NAD^+^ metabolism in the liver, heart, kidney and lung from female wistar rats aged from 3 to 24 months, spanning life stages from young adulthood to old age [36]. We quantified the levels of oxidative stress (in the form of protein carbonyls, lipid peroxidation, and oxidative DNA damage), total antioxidant and NAD^+^ levels and PARP, Sirt1 and mitochondrial activities in these tissues at different stages of life. Our results suggest that oxidative stress induced NAD^+^ depletion could play a significant role in the aging process, by compromising, energy production, DNA repair and genomic surveillance.

## Materials and Methods

### Reagents and Chemicals

Phosphate buffer solution (PBS) was from Invitrogen (Melbourne, Australia). Nicotinamide, bicine, β-nicotinamide adenine dinucleotide reduced form (β-NADH), 3-[-4,5-dimethylthiazol-2-yl]-2,5-diphenyl tetrazolium bromide (MTT), alcohol dehydrogenase (ADH), sodium pyruvate, TRIS, γ-globulins, N-(1-naphthyl) ethylenediamine dihydrochloride, EGTA, EDTA, tricarboxylic acid (TCA), Hepes, proteinase K, Percoll, mannitol, 1,-dithio DL-threitol (DTT), KCN, decylubiquinone, succinate, antimycin, rotenone, cytochrome *c*, and sodium borohydride were obtained from Sigma-Aldrich (Castle-Hill, Australia). Phenazine methosulfate (PMS) was obtained from ICN Biochemicals (Ohio, USA). Bradford reagent was obtained from BioRad (Hercules, CA, USA). DAPI and polyclonal antibodies (pAb) for β-actin and all chemicals used for Western blots (unless otherwise stated) were obtained from Sigma-Aldrich (Castle-Hill, Australia). Polyclonal antibodies for detection of (E)-4- Hydroxynonenal, Sirt1, phospho-H2AX-ser139 were obtained from Alexis Biochemicals (San Diego, CA, USA). Monoclonal antibody for the detection of Poly(ADP-ribose) was purchased from Alexis Biochemicals (San Diego, CA, USA). Polyclonal antibody for the detection of acetylated p53 was obtained from Abcam (Cambridge, UK). Monoclonal antibody to total p53 was obtained from Millipore (Melbourne, Australia). Alexa 488- or Alexa 594-conjugated anti-mouse IgG or anti-rabbit were purchased from Invitrogen. All commercial antibodies were used at the concentrations recommended by the manufacturer.

### Animals

Female wistar rats were used and experiments were designed to target the following age groups: 3 months old (equivalent to a young human adult aged 20 years), 12 month old (equivalent to a middle-aged human aged 40 years) and 24 month old (equivalent to an aged human greater than 80 years) [37]. The animals were individually housed in an environmentally controlled room under a 12∶12 hour light/dark cycle at 23°C and were given commercial rat chow and water *ad libitum*. All experiments were performed according to the Animal Ethics Committee of the University of Sydney. Anaesthesia was induced with a mixture of O_2_, NO_2_, and 5% halothane, and then maintained by an intraperitoneal injection of sodium pentobarbitone (60 mg kg^−1^). Transcardial perfusion was performed using 0.1 M DPBS, pH 7.4. Whole heart, lung, liver and kidney, were removed, washed with DPBS and used immediately for a variety of biochemical and histochemical procedures.

### Assay of *o-* and *m-* tyrosine for the Measurement of Protein Carbonyl Formation

The assay for *o-* and *m-* tyrosine was performed as previously described [38]. Briefly, calibration standards of phenylalanine (313 pmol and 50 nmol) and *o-* and *m-* tyrosine (313 fmol to 50 pmol) were used for quantification. Labelled [^13^C_6_]-phenylalanine was used as an internal standard and was added to all samples and standards. The liver, heart, kidney and lung were placed in tapered glass vial. The protein was then allowed to precipitate (∼18 h, −20°C) following the addition of 10 volumes of acetone/HCl (100∶1, v∶v). The precipitate was centrifuged (14,000 g, 30 min, ambient temperature) and the supernatant discarded. Internal standard (10 µl, 1 mg/ml [^13^C_6_]-phenylalanine) containing trace quantities of [^13^C_6_]-tyrosine, was added to all samples and standards, and dried under reduced pressure (<1 Torr, 1–2 h). Afterwards, gas phase acid hydrolysis was performed at 150°C for 1 h. Samples and standards were then derivatised using a three-step derivatisation approach, using heptafluorobutyric anhydride (HFBA), pentafluorobenzylbromide (PFBBr) and N,O-bis(trimethylsilyl)-trifluoroacetamide (BSTFA), vacuum dried for 10 min, and reconstituted in 50 µl ethyl acetate. Each standard and sample (1 µl) was injected into the GC/MS using pressure pulse splitless loading (6890N gas chromatograph interfaced to 5973 mass selective detector; Agilent technologies, Ryde, Australia), with methane as the ECNI reagent gas. Chromatography was performed on a fused silica capillary column (HP-5MS; 30 m×0.25 mm i.d.×0.25 µm, film thickness), with helium carrier gas and using the following chromatographic parameters: inlet temperature 250°C, transfer line temperature 280°C, programmed oven temperature gradient with initial temperature of 150°C for 3 min, then a temperature ramp of 30°C/min to 290 and a final time of 3 min at 290°C. Final *o-* and *m-* tyrosine levels were expressed relative to phenylalanine levels.

### Western Blots for the Detection of 4-Hydroxynonenal, Poly(ADP)-ribose, Sirt1, and Total/Acetylated p53 Protein Expression

The whole liver, heart, kidney and lung were homogenised in RIPA lysis buffer containing 50 mM Tris-HCl (pH 7.4); IGEPAL 1%; 0.25% Na-deoxycholate; 1 mM EDTA, 150 mM NaCl; 1 µg/ml each of aprotinin, leupeptin and pepstatin; 1 mM Na_3_VO_4_; and 1 mM NaF. After 1 h, the homogenate was obtained by centrifuging at 14,000 g, for 30 min at 4°C. Protein concentration was determined using the Bradford protein assay. Equal amounts of protein extract (30 µg) were dissolved in Laemmli sample buffer (Hercules, CA, USA), boiled for 5 min, electrophoresed on 8–12% (v/v) polyacrylamide SDS-PAGE gels (BioRad, Hercules, CA, USA), and electrotransferred onto PVDF membranes (BioRad, Hercules, CA, USA). Membranes were blocked with 5% non-fat milk dissolved in TBS for 1 h and incubated with primary antibody overnight at 4°C. The primary antibodies used are described in Table 1. After incubation with primary antibodies, membranes were washed in TBS-Tween-20 and incubated with HRP conjugated secondary antibodies (Sigma, Castle Hill, Australia) for 1 h at room temperature. After further washing in TBS-Tween-20, the membranes were incubated with an ECL plus reagent (RPN2132, Amersham) and protein bands were visualised on X-ray films. The bands were quantified by ImageJ software, and normalised to β-actin, which served as an internal control.

**Table 1:** List of primary antibodies used.

Antibody	Type	Antigen	Dilution	Source
**(E)-4-Hydroxynonenal**	Polyclonal	Free HNE (E)-4-hydroxynonenal	1∶1000	Alexis Biochemicals
**Phospho-H2AX-Serine139**	Polyclonal	Phosphorylated H2AX at Serine 139	1∶1000	Alexis Biochemicals
**Poly(ADP-ribose) (10H)**	Monoclonal	Poly(ADP-ribose)	1∶400	Alexis Biochemicals
**Sirt1**	Polyclonal	Sirt1	1∶2000	Alexis Biochemicals
**Acetyl K386**	Polyclonal	Acetylated p53 at lysine 386	1∶1000	Abcam
**p53 Oncogene**	Monoclonal	Total p53 oncogene	1∶1000	Millipore

### Total Antioxidant Capacity Assay

The total antioxidant capacity in aging liver, heart, kidney and lung was evaluated by Trolox equivalent antioxidant capacity assay using a standard antioxidant assay kit (Cayman, Michigan, USA). Briefly, the tissue was homogenised on ice in a buffer containing 5 mM potassium phosphate; 0.9% NaCl; and 0.1% glucose, pH 7.4. The samples were centrifuged at 10,000 g for 15 min at 4°C, and the supernatant was collected for the assay. Briefly, 10 µl of sample was added to 10 µl of Metmyoglobin and 150 µl of Chromogen. The reaction was initiated by adding 40 µl of hydrogen peroxide working solution. The samples were incubated on a shaker for 5 min at room temperature and the absorbance was read at 405 nm using the Model 680XR microplate reader (BioRad, Hercules). The absorbance values obtained for the samples were compared with a standard curve obtained using Trolox (6-hydroxy-2,5,7,8-tetramethyl-chroman-2-carboxylic acid), a permeable cell derivative of vitamin E commonly employed as an antioxidant. The results were expressed as mmol Trolox/L/mg protein.

### DNA Damage Assay

Since H2AX phosphorylation at serine 139 correlates very closely with each double-stranded DNA break, phosphor-H2AX is a sensitive marker for DNA damage [39]. We measured phosophorylation of H2AX at serine 139 using a DNA damage assay kit (Active Motif, Carlsbad, California, USA). Briefly, the liver, heart, kidney and lung was suspended on ice in a buffer containing 1 mM PMSF and pelleted at 10,000 g for 4 min at 4°C. Afterwards 200 µl of warm SDS lysis buffer containing 1 µg/ml each of aprotinin, leupeptin and pepstatin and 1 mM PMSF were then added and incubated for 10 min on ice. All samples were sonicated to generate 100 - to 1000-bp DNA fragments. 5 µg/ml of anti-phospho-H2AX-ser139 was added to the lysate with cold DPBS and allowed to incubate overnight at 4°C. The primary antibody was removed by washing the lysate 3 times with 200 µl DPBS. Alexis 488 goat anti-rabbit IgG secondary antibody (1∶1000) was added to the lysate and incubated for 1 hour at room temperature. The secondary antibody was removed by washing the lysate twice with 200 µl DPBS. The fluorescence was read using Fluostar Optima Fluorometer (NY, USA). Filter excitation and emission was set at 485 nm and 520 wavelengths respectively.

### Isolation and Extraction of Nuclei for PARP and Sirt1 deacetylase Activity Assays

Aliquots of homogenate from the liver, heart, kidney and lung (without protease inhibitors) were spun through 4 ml of 30% sucrose solution containing 10 mM Tris HCl (pH 7.4); 10 mM NaCl; and 3 mM MgCl_2_ at 1,300 g for 10 min at 4°C. The remaining pellet was washed with cold 10 mM Tris-HCl (pH 7.4) containing 10 mM NaCl. The nuclei was later suspended in 50–100 µl extraction buffer containing 50 mM Hepes KOH (pH 7.4); 420 mM NaCl; 0.5 mM EDTA; 0.1 mM EGTA; and glycerol 10%, sonicated for 30 s, and allowed to stand on ice for 30 min. After centrifugation at 10,000 g for 10 min, an aliquot of the supernatant was used to determine protein concentration using the Bradford protein assay.

### PARP Activity Assay

PARP activity was measured in nuclear extracts from the liver, heart, kidney and lung of young, middle-aged, and aged rats, using a new operational protocol relying on the chemical quantification of NAD^+^ modified from Putt et al. [40]. The final reaction mixture contained 10 mM MgCl_2_, Triton X-100 (1%), and 20 µM NAD^+^ in 50 mM Tris buffer, pH 8.1. The plate was then incubated for 1 hour and the amount of NAD^+^ consumed was measured by the NAD(H) microcycling assay using the Model 680XR microplate reader (BioRad, Hercules). The results were expressed as NAD^+^ consumed/h/mg protein.

### Sirt1 deacetylase Activity

Sirt1 deacetylase activity was evaluated in nuclear extracts from the liver, heart, kidney and lung of young, middle-aged, and aged rats, using the Cyclex SIRT1/Sir2 Deacetylase Flourometric Assay Kit (CycLex, Nagano, Japan). The final reaction mixture (100 µl) contained 50 mM Tris-HCl (pH 8.8), 4 mM MgCl2, 0.5 mM DTT, 0.25 mA/ml Lysyl endopeptidase, 1 µM Trichostatin A, 200 µM NAD^+^, and 5 µl of nuclear sample. The samples were mixed well and incubated for 10 min at room temperature and the fluorescence intensity (ex. 340 nm, em. 460 nm) was measured every 30 s for a total of 60 min immediately after the addition of fluorosubstrate peptide (20 µM final concentration) using Fluostar Optima Fluorometer (NY, USA) and normalised by the protein content. The results are reported as relative fluorescence/µg of protein (AU).

### Measurement of Intracellular NAD^+^/NADH Levels

Total intracellular NAD (NADH+NAD^+^) concentration was measured spectrophotometrically using the thiazolyl blue microcycling assay established by Bernofsky and Swan (1973) adapted for 96 well plate format by Grant and Kapoor (1998) [41], [42]. Briefly, each assay contained 100 mM bicine, pH 7.8; 0.42 mM MTT, and 1.66 mM PMS. For NAD^+^ measurement, 20 µl of ADH in 0.15% ethanol was added to the reaction mixture. The amount of NAD and NADH were measured as the change in absorbance at 590 nm at 37°C for 10 minutes with a Model 680XR microplate reader (BioRad, Hercules). The ratio of NAD^+^/NADH was calculated based on results of NAD^+^ and NADH concentrations.

### Isolation of Mitochondria

All procedures were carried out at 0–4°C. Briefly, the liver, heart, kidney and lung were excised, washed with DPBS, and treated with proteinase K (1 mg/ml) for 30 s, washed with buffer A (250 mM mannitol; 0.5 mM EGTA; 5 mM Hepes; and fatty acid free bovine serum albumin 0.1%, pH 7.4 at 4°C). The samples homogenised with buffer A using a Teflon pestle. The homogenate was centrifuged twice at 600 g for 5 min at 4°C. The supernatants were mixed and centrifuged at 10,300 g for 10 min at 4°C. The mitochondrial pellets were suspended in 0.5 ml buffer A and transferred to ultracentrifuge tubes containing 1.4 ml buffer B (225 mM mannitol; 1 mM EGTA; 25 mM Hepes; and fatty acid free bovine serum albumin (BSA) 0.1%, pH 7.4 at 4°C) and 0.6 ml Percoll. The mixture was centrifuged at 105,000 g for 30 min at 4°C. The pure mitochondrial fraction was purified by washing twice with buffer A at 10,300 g for 10 min at 4°C to remove the Percoll and frozen to −80°C. An aliquot was used to determine the mitochondrial protein content using the Bradford protein assay.

### Determination of Mitochondrial Complexes I, II, III, and IV activities

To determine the complex I activity, submitochondrial fractions (0.6 mg/ml) were incubated for 3 min in buffer solution containing 250 mM sucrose; 50 mM potassium-phosphate; 1 mM KCN; 50 µM decylubiquinone; 0.8 µM antimycin, pH 7.4. The reaction was started following the addition of NADH (100 µM). The activity of NADH CoQ oxidoreductase was measured as the rate of oxidation of NADH at 340 nm using the Model 680XR microplate reader (BioRad, Hercules). The activity of complex I was expressed as nmol oxidised NADH/min/mg protein. The activity of complex II was measured in buffer solution containing submitochondrial fractions (0.03 mg/ml); 100 mM potassium-phosphate; 20 mM succinate; 0.8 µM antimycin; 50 µM rotenone; 2 µM KCN; 50 µM DCIP, pH 7.4. The reaction was initiated by the addition of 50 µM decylubiquinone. The activity of succinate:DCIP oxireductase was measured as the rate of reduction of 2, 6-DCIP at 600 nm with 520 nm as reference wavelength. The activity of complex II was expressed in nmol reduced DCIP/min/mg protein. The activity of complex III was measured in buffer solution containing submitochondrial fractions (0.03 mg/ml); 35 mM potassium-phosphate; 5 mM MgCl_2_; 2.5 mg/ml BSA; 50 mM rotenone; 1.8 mM KCN; 2 mM decylubiquinone, pH 7.5. The reaction was initiated by the addition of 125 µM cytochrome *c*. The activity of ubiquinol:cytochrome *c* reductase was measured as the rate of reduction of cytochrome *c* at 550 nm with 580 nm as the reference wavelength. The activity of complex III was expressed in nmol reduced cytochrome *c*/min/mg protein. The activity of complex IV was measured in a buffer solution containing submitochondrial fractions (0.1 mg/ml); 50 mM potassium-phosphate, pH 6.8. The reaction was started by the addition of 75 µM cytochrome *c* previously reduced with sodium borohydride and measuring the absorbance at 550 nm. The activity of cytochrome *c* oxidase was expressed as nmol oxidised cytochrome *c*/min/mg protein.

### Immunoflourescence Staining for 4-Hydroxynonenal, Phospho-H2AX-Serine139, Poly(ADP)-ribose, and Sirt1

Liver, heart, kidney and lung whole mounts were immersion-fixed with ice cold 70% ethanol for 20 mins followed by 4% paraformaldehyde (PFA), pH 7.4 for 10 min at 4°C. Immunostaining was established on brain whole mount. Fixed tissue were permeabilised with 1% Triton-X 100 in DPBS for 30 min at room temperature and non-specific binding was blocked with 1% BSA in DPBS for 2 h before application of primary antibodies. All specific primary mAb or pAb antibodies were diluted in 1% BSA in PBS and incubated overnight at 4°C. Tissue whole mounts were washed three times with DPBS and incubated for 1 h at 37°C with the appropriate labeled secondary antibodies (goat anti-mouse IgG or goat anti-rabbit IgG coupled to Alexa 488 or Alexa 594). Nuclear staining was performed using DAPI at 1 µg/ml for 5 min at room temperature. The slides were washed 3 times in DPBS at room temperature and coverslips were mounted on glass slides with Flouromount-G and were examined with an Olympus BX60 fluorescence microscope fitted with a SensiCam digital camera. Titration series and conjugate experimental controls were performed on both primary and secondary antibodies to optimise for low background noise, maximal stain sensitivity, avoidance of non-specific staining and cross-reactivity.

### Bradford Protein Assay for the Quantification of Total Protein

DNA damage, total antioxidant capacity, PARP and Sirt1 activities, NAD^+^ concentration, and mitochondrial function were adjusted for variations in protein number using the Bradford protein assay described by Bradford [43].

### Data Analysis

Results obtained are presented as the means ± the standard error of measurement (SEM) of at least eight animals per age group analysed in duplicate. One way analysis of variance (ANOVA) and post hoc Tukey's multiple comparison tests were used to determine statistical significance between treatment groups. Differences between treatment groups were considered significant if p was less than 0.05 (p<0.05).

## Results

### Age-related Increase in Protein Carbonyl Formation

Hydroxyl radical attack on the amino acid phenylalanine generates *o-*, *m-* and *p-* tyrosine were detected using gas chromatography/mass spectrometry (GC/MS) [44], [45]. Figure 1 shows the age-related changes in *o*- (Fig. 1A) and *m-* tyrosine (Fig. 1B) levels in the liver, heart, kidney and lung. Our results show a significant increase in both *o- and m*- tyrosine formation with age, with the highest rate of increase occurring after 12 months of age in all organs (p<0.01).

**Figure 1:** Increased formation of oxidatively modified proteins in the liver, heart, kidney, and lung with age. Increased levels of (A) *o-* tyrosine and (B) *m-* tyrosine were reported in the brain after 12 months of age compared to 3 month old rats. All values are means ± S.E from tissue obtained from eight different rats for each age group. Significance ^*^p<0.01 compared to 3 month old rats.

### 4-HNE as a Biomarker for Lipid Peroxidation in Aging

Peroxidative damage to cellular lipid constituents was determined by using 4-HNE as a marker of lipid peroxidation. Increased 4-HNE protein expression using western blotting was observed in the liver (p<0.01) (Fig. 2A), heart (p<0.01) (Fig. 2B), kidney (p<0.01) (Fig. 2C) and lung (p<0.01) (Fig. 2D), consistent with an increase in protein carbonyl formation (Fig. 1).Using immunohistofluorochemistry, we stained frozen sections for 4-HNE (Fig. 2E). Two age related changes are clearly visible: (1) There is an increase in 4-HNE expression consistent with the previous western blot studies (Fig. 2A–D). (2) Aged tissue appears to demonstrate significantly lower cell volume, indicative of extensive cell loss occurring during the aging process.

**Figure 2:** Increased oxidative damage to lipids in selected brain regions with age. (A) Liver, (B) heart, (C) kidney, and (D) lung were analysed by Western blotting using anti-4HNE antibody. The blots shown are representative tracings of an experiment done eight times. Graphs are mean ± S.E from tissue obtained from eight different rats for each age group. Each bar of the quantification graph represents the corresponding band for each age group. Significance ^*^p<0.01 compared to 3 month old rats. (E) Immunodetection of 4-HNE in the liver, heart, kidney, and lung from 3 month, 12 month and 24 month old rats. 4-HNE (green) and DAPI (blue). Higher immunoreactivity for 4-HNE was observed in 12 and 24 month old rats compared to 3-month old rats.

### Total Antioxidant Capacity Declines with Aging

To investigate changes in endogenous antioxidant function age, we measured total antioxidant capacity *in-situ* using the Trolox assay. We observed a significant reduction in total antioxidant activity by 12 months of age in all organs with the most rapid decline occurring between 12 and 24 months (p<0.01) (Fig. 3).

**Figure 3:** Total antioxidant capacity significantly declined in the rat liver, heart, kidney, and lung with age. All values are means ± S.E from tissue obtained from eight different rats for each age group. Significance ^*^p<0.01 compared to 3 month old rats.

### DNA Damage Increases with Aging

The aging process is also considered to cause changes in the DNA repair process leading to increased vulnerability to DNA damage [7]. We assessed DNA damage by measuring the phosphorylation of H2AX at Serine139 residue using a flourometric assay. Increased DNA damage was observed in all aged organs assessed in this study by 12 months of age with accelerated damage occurring between 12 and 24 months (Fig. 4) (p<0.01). Immunohistofluorochemistry (Fig. 4C) confirmed the increase in phospho-H2AX-Serine139.

**Figure 4:** Increased DNA damage was reported in the rat liver, heart, kidney, and lung with age. (A) DNA damage was determined by measuring the flourescence of phosphorylated H2AX at Serine139 using the Fluostar Optima Fluorometer (NY, USA). All values are means ± S.E from tissue obtained from eight different rats for each age group. Significance ^*^p<0.01 compared to 3 month old rats. (B) Immunodetection of phosphor-H2AX-Serine139 in the liver, heart, kidney, and lung from 3 month, 12 month and 24 month old rats. Phosphor-H2AX-Serine139 (green) and DAPI (blue). Higher immunoreactivity for phosphor-H2AX-Serine139 was observed in 12 and 24 month old rats compared to 3-month old rats.

### PARP Activation & Poly(ADP-ribose) polymers

To demonstrate a direct link between DNA damage and poly-ADP-ribosylation, we measured PARP activity in nuclei from the liver, heart, kidney and lung of aging rats. Our results show a significant (p<0.01) up-regulation of PARP activity in all organs by 12 months of age (Fig. 5A). This is consistent with increased formation of poly(ADP-ribose) nuclear protein in the liver (Fig. 5B), heart (Fig. 5C), kidney (Fig. 5D),and lung (Fig. 5E), using western blot and immunohistofluorochemistry (Fig. 5F).

**Figure 5:** Increased Poly(ADP-ribose) activity in the brain with age. (A) PARP activity was determined in aging tissue using a spectrophotometric assay. All values are means ± S.E from tissue obtained from eight different rats for each age group. Significance ^*^p<0.01 compared to 3 month old rats. (B) Western blotting for poly(ADP-ribose) in (i) liver, (ii) heart, (iii) kidney, and (iv) lung with aging using anti-Poly(ADP-ribose) (10H) antibody. The blots shown are representative tracings of an experiment done eight times. Graphs are mean ± S.E from tissue obtained from eight different rats for each age group. Each bar of the quantification graph represents the corresponding band for each age group. Significance ^*^p<0.01 compared to 3 month old rats. (C) Immunodetection for poly(ADP-ribose) in the liver, heart, kidney and lung from 3 month, 12 month and 24 month old rats. Poly(ADP-ribose) (green) and DAPI (blue). Higher immunoreactivity for poly(ADP-ribose) was observed in 12 and 24 month old rats compared to 3-month old rats.

### Intracellular NAD^+^(H) Levels

As NAD^+^ is the sole substrate for PARP we assessed the impact of PARP activation on intracellular NAD^+^ content in the same aging rat tissue. We found that increased PARP activity was associated with a significant (p<0.01) reduction in the NAD^+^ content by 24 months of age in each of the organs investigated (Fig. 6A). This is in line with a significant increase in NADH (Fig. 6B) (p<0.01) and a significant decline in the NAD^+^∶NADH ratio (Fig. 6C) (p<0.01). Most of the decline in intracellular NAD^+^ content was observed after 12 months of age, and appears to be more noteworthy in the heart.

**Figure 6:** Increased PARP activation alters pyridine nucleotide metabolism with aging. (A) NAD^+^ content and (B) NADH content were determined in the rat liver, heart, kidney and lung with aging using a spectrophotometric assay. All values are means ± S.E from tissue obtained from eight different rats for each age group. Significance ^*^p<0.01 compared to 3 month old rats. (C) NAD^+^∶NADH ratio was determined as the total NAD^+^ content divided by total NADH levels. All values are means ± S.E from tissue obtained from eight different rats for each age group. Significance ^*^p<0.01 compared to 3 month old rats.

### Sirt1 deacetylase Activity (but not protein levels) Declines with Aging

Sirt1 is localised in the nucleus [27]. Therefore, both Sirt1 protein level and activity were measured in the liver, heart, kidney and lung of aging rats. Aging induced a significant decline in Sirt1 activity in the liver (p<0.01), heart (p<0.01), kidney (p<0.01), and lung (p<0.01) (Fig. 7A) consistent with decreased substrate (NAD+) availability (Fig. 6). In contrast, we observed that aging significantly (p<0.01) increased the amount of Sirt1 protein in the nucleus in all organs examined in this study, using both western blotting (Fig. 7B–E) and immunohistofluorochemistry (Fig. 7F).

**Figure 7:** Reduced NAD^+^ levels contributes to reduced Sirt1 activity in the liver, heart, kidney and lung with aging. (A) Reduced Sirt1 activity was observed in the rat liver, heart, kidney and lung after 12 months of age using a flourometry. All values are means ± S.E from tissue obtained from eight different rats for each age group. Significance ^*^p<0.01 compared to 3 month old rats. (B) Western blotting for Sirt1 in (i) liver, (ii) heart, (iii) kidney, and (iv) lung with aging using anti-Sirt1 antibody. The blots shown are representative tracings of an experiment done eight times. Graphs are mean ± S.E brains from tissue obtained from eight different rats for each age group. Each bar of the quantification graph represents the corresponding band for each age group. Significance ^*^p<0.01 compared to 3 month old rats. (C) Immunodetection for Sirt1 in the liver, heart, kidney and lung from 3 month, 12 month and 24 month old rats. Sirt1 (red) and DAPI (blue). Higher immunoreactivity for Sirt1 was observed in 12 and 24 month old rats compared to 3-month old rats.

### Increased p53 Acetylation in Aging Brain

To confirm the effect of decreased NAD^+^ levels and Sirt1 function on the acetylation status of p53, we measured both acetylated and total p53 protein levels using western blotting. As shown in Figure 8, we found a significant age-dependent increase in acetylated p53 expression in the liver (p<0.01), heart (p<0.01), kidney (p<0.01), and lung (p<0.01). However, no change was observed in total p53 content between young and aged rats in all organs investigated.

**Figure 8:** Reduced Sirt1 activity induces p53 acetylation in the liver, heart, kidney and lung with aging. Acetylated p53 and total p53 levels were determined by Western blotting in (A) liver, (B) heart, (C) kidney, and (D) lung with aging using anti-acetylated p53 and anti-total p53 antibodies. The blots shown are representative tracings of an experiment done eight times. Graphs are mean ± S.E brains from tissue obtained from eight different rats for each age group. Each bar of the quantification graph represents the corresponding band for each age group. Significance ^*^p<0.01 compared to 3 month old rats.

### Impaired Mitochondrial Respiratory Chain Activity with Aging

Although mitochondrial production of ROS has been shown to increase with advancing age [46], changes in the mitochondrial redox status with age in the heart, lung, liver and kidney has not, to our knowledge, been evaluated. We measured the activities of the mitochondrial respiratory complexes as shown in Figure 9A–D. The activity of all complexes decreased after 12 months of age, and reached statistical significance at 24 months in the liver (p<0.01), heart (p<0.01), kidney (p<0.01) and lung (p<0.01). Fig. 8E shows the ATP levels determined in all organs during the aging process. ATP levels significantly (p<0.01) declined in the heart, lung, liver and kidney after 12 months of age. This is in line with increased PARP activation and decline in cellular NAD^+^ content during the aging process.

**Figure 9:** Oxidative stress-mediated reduction in mitochondrial respiratory chain activity in the liver, heart, kidney and lung with age. Reduced (A) complex I, (B) complex II, (C) complex III, and (D) complex IV, activities at 24 months of age. All values are means ± S.E from tissue obtained from eight different rats for each age group. Significance ^*^p<0.01 compared to 3 month old rats.

## Discussion

There is growing consensus around the hypothesis that oxidatively damage proteins, lipids, and nucleic acids play a key role in the aging process. Oxidative stress occurs in several degenerative diseases including neurodegenerative disease (e.g. Alzheimer's, Parkinson's), rheumatoid arthritis, atherosclerosis, diabetes, and cardiovascular disease [47]. This study is the first to investigate the impact of age associated changes in oxidative stress levels on both intracellular NAD^+^ levels and activity of the ‘longevity’ enzyme Sirt1. This study is also the first to report changes in *o-* and *m-* tryosine (specific markers of protein oxidation) in aging heart, lung, liver and kidney.

In this report we provide consistent evidence of accumulating oxidative damage to tissue proteins, lipids and nuclear DNA with age. Reactive oxygen species (ROS) are byproducts of normal cellular physiology [48]. A delicate balance between ROS generation and detoxification is maintained by several cellular antioxidant defense systems [49], [50]. These comprise antioxidant enzymes such as SOD1, catalase, glutathione peroxidase; and endogenous non-enzymatically acting compounds, such as vitamins A, C and E [9]. Nevertheless, various endogenous and exogenous triggers may stimulate the overproduction and accumulation of ROS leading to oxidative damage [9]. While oxidative stress increases with aging, it is yet unclear at which age free-radicals may act to initiate the senescence process. Young and aged rat models are relatively homogenous in their gene expressions in the various organs. This may be in contrast to young adult and aged human populations which may demonstrate much greater heterogeneity. Unlike aged rodents, humans may diverge in their rates of aging, as they translate from middle age to old age. In this study at middle age (i.e.12 months), female wistar rats already exhibit higher levels of oxidative stress induced damage to proteins, lipids, and DNA, with a lower total antioxidant efficiency than young adult animals of 3 months of age. Our results suggest an age-dependent increase in oxidative stress in these organs that appears to accelerate after middle age (i.e.12 months). These data support the existence of a progressive disequilibrium between the formation of ROS and the antioxidant protective mechanisms during the process of normal aging [9] in rats that may be applicable to the human population.

Apart from increased levels of protein oxidation and lipid peroxidation, DNA is also susceptible to oxidative damage by ROS [7]. We assessed DNA damage by measuring the phosphorylation of histone H2AX at Serine139 residue. H2AX phosphorylation is considered a specific reporter of double-stranded DNA damage [39]. The level of DNA damage increased with age in all organs consistent with an increase in protein carbonyls and lipid peroxidation. Experimental data from other laboratories have shown a similar increase in DNA damage, (e.g. 8-oxoguanine) in the heart, lung, liver and kidney of aging rats [51].

The DNA damage associated with oxidative stress is known to activate the NAD^+^-dependent DNA repair enzyme, PARP, which assists in combination with the enzymes of the base-excision-and-repair complex of the cell in energy-consuming repair processes [12], [52], [53]. The vital role of PARP activation in several diseases has been obtained from experimental studies using PARP inhibitors, PARP knock-down mice, and clinical trials. Recent studies have shown the protective effects of PARP inhibitors on ischaemic heart and liver, diabetic kidney disease, and endotoxin-induced acute lung injury, arguably due to the preservation of NAD^+^ levels [20], [21], [22], [23], [24]. PARP activation can also promote apoptosis by stabilising p53, and mediating the translocation of apoptosis-inducing factor from mitochondria to the nucleus [19], [54]. Several lines of evidence reported here show that PARP activation increases in the aging heart, lung, liver, and kidney (Fig. 5), and depletes cellular NAD^+^ levels (Fig. 6). Theoretically this should lead to a reduction in Sirt1 deacetylase activity and accumulation of acetylated p53. Consistent with this prediction we observed that increased PARP activation (Fig. 5) was associated with NAD^+^ depletion (Fig. 6) which was accompanied by a decrease in Sirt1 deacetylase activity (Fig. 7).

It is well established that genotoxic stress can kill cells by depleting the intracellular NAD^+^ pools due to extensive use of NAD^+^ as a substrate for PARP [12], [13], [16], [19]. Results from the present study, consistent with others, suggests that both PARP and Sirt1 compete for the same limiting intracellular NAD^+^ pool [55]. One study showed that PARP activation depleted intracellular NAD^+^ levels and reduced Sirt1 deacetylase activity in DNA damaged in cardiac myocytes [55]. Replenishing intracellular NAD^+^ levels by increasing NAD^+^ levels was able to restore cellular viability but only in the presence of functional Sirt1 [55]. As NAD^+^ serves as a cofactor for key glycolytic and mitochondrial enzymes, vulnerable cells subsequently lose their ability to carry out energy dependent functions including the maintenance of cell wall integrity and DNA/RNA synthesis and consequently die [56]. We demonstrated, for the first time, that aging in the rat is associated with decreased tissue levels of NAD^+^. This may lower the rate of cell survival in response to several endogenous and exogenous stressors. As NAD^+^ is the only substrate for both PARP and Sirt1 activities, maintaining optimal NAD^+^ content is crucial to counteract the age-related degeneration observed during the aging process [56], [57].

As a substrate for the sirtuin family of NAD^+^ dependent deacetylases, known as silent information regulators of gene function [27]. This discovery suggests that gene silencing by this system might be related to metabolic rate and hence to NAD^+^ concentrations, whose levels therefore may be directly proportional to a longer lifespan [28]. While several studies have demonstrated the protective roles of sirtuin activators during aging [30], [34], [35], [58], [59], [60], [61], [62], [63], little is known regarding role of Sirt1 in the aging heart, lung, liver, and kidney.

The present results show that aging increases the amount of available Sirt1 protein and activities of Sirt1 in nuclear extracts in the heart, lung, liver, and kidney. The activity per molecule of Sirt1 appears to become lower in these organs as the animal ages, suggesting the presence of more inactive or less active molecules in aged animals. These observations are in line with a previous study which reported a decrease in Sirt1 activity but not Sirt1 protein expression in skeletal muscle of aged rats [64].Two possibilities, which are not mutually exclusive, may explain this observation: 1) Oxidative damage may potentially inhibit Sirt1 activity in a similar way to several other proteins [65] and/or 2) It is also likely that the age-associated drop in NAD^+^ content due to increased demand by PARP in the DNA repair process limits the Sirt1 substrate NAD^+^ thereby limiting Sirt1 activity. A compensatory mechanism which increases the production of the Sirt1 protein [64] would increase its relative success when competing for the limited NAD^+^ pool.. Sirt1 deficiency has been shown to accentuate apoptosis of renal medullary cells [66] and cardiac mycocytes [55]. Over-expression of Sirt1 has been shown to promote the resistance of these cells to oxidative insult, both *in vitro* and *in vivo* [67]. The protective function of Sirt1 has been reported in other organs such as the heart, neurons, lung, liver [67], [68], [69], [70]. Given the pivotal role of Sirt1 as an anti-stress and anti-aging protein, targeting Sirt1 by either Sirt1 activators or increasing its substrate (i.e. NAD^+^) availability may prove therapeutically beneficial for the prevention of age-related cardiovascular, respiratory, hepatic, and renal dysfunction.

Because Sirt1 activity is affected by the NAD^+^∶NADH ratio [71], we determined the NAD^+^ and NADH content in aging heart, lung, liver, and kidney. Our results show a significant decline in the NAD^+^∶NADH ratio with aging, consistent with a decline in NAD^+^ levels and an increase in NADH levels. This indicates that age related metabolic changes may influence NAD^+^ and NADH upstream of Sirt1 similar to what was observed in yeast Sir2α and in the skeletal muscle [71].

To examine the downstream effect of Sirt1 deacetylase activity in cellular processes, we measured the expression of both total and acetylated p53 in aging rat tissue. The main tumour suppressor protein, p53 regulates the expression of several gene products that either lead to cell cycle arrest in G1 phase and prevent DNA replication immediately before the repair of damage, or cause cell death via an apoptotic mechanism [72]. We observed a significant increase in acetylated p53 protein while no change was observed in total p53 protein in all organs was apparent. Higher acetylation levels of p53 have been reported in cardiac myocytes following treatment with the oxidant H_2_O_2_, probably resulting from decreased NAD^+^ and impaired Sirt1 deacetylase activity [55]. A recent report showed that microRNA 34a (miR-34a), a tumour suppressor gene inhibiting Sirt1 expression also increases acetylated p53 levels, thus stimulating transcriptional targets of p53 responsible for promoting cell-cycle arrest, and apoptosis [73]. While p53 has been shown to be bind to PARP and be poly(ADP-ribosylated), an effect which enhances their pro-apoptotic activity, Sirt1-dependent deacetylation inhibits their apoptotic activity [55]. These results suggest that changes in intracellular NAD^+^ levels may regulate the post-translational acetylation of p53, thus providing further evidence of the association between NAD^+^ levels, oxidative DNA damage-mediated PARP activation, and reduced Sirt1 deacetylase activity [55].

One factor which may sensitise cells to increased DNA damage is impaired mitochondrial function [74]. The mitochondrial electron transport system can trigger the formation of superoxide leading to increased production of H_2_O_2_ by superoxide dismutase [49], [50]. Reduced electron flow through the mitochondrial respiratory chain, particularly through the inhibition of complex I or complex III, favours the enhanced production of superoxide and H_2_O_2_ [75]. Together, with the age-dependent increase in oxidative stress and decline in NAD^+^ and ATP content, we found a tendency to the reduction in the activity of the respiratory complexes with age in all organs. Sipos et al. (2003) showed that mitochondrial formation of H_2_O_2_ due to complex I inhibition is more clinically relevant than ROS production due to inhibition of complex III and IV *in situ* [76]. Using the same experimental paradigm, Rodriguez et al. (2008) reported similar mitochondrial oxidative failure in the diaphragm of senescent prone mice [49].

It has also been demonstrated that an increased NADH∶NAD^+^ ratio, favours ROS generation by the catalytic activity of α-Ketoglutarate dehydrogenase (α KGDH) [77]. The dependence on ROS production by α KGDH on the intracellular NADH content may play a crucial role in promoting the accumulation of free radicals in aging. When the reoxidation of NADH is impaired due to reduced complex I activity, the NADH∶NAD^+^ ratio increases, thus reducing the activity of several NAD^+^ dependent dehydrogenases [77]. Moreover, NADH is also able to promote the formation of H_2_O_2_ in the presence of iron [78]. Given the observations in the present study, increased ROS production in aging may be a consequence of impaired mitochondrial respiratory function, and may, at least in part, be attributed to increased NADH∶NAD^+^ ratio inducing free radical production via αKGDH and Fenton chemistry.

Overall, our results show that oxidative stress increased with age, (appearing to accelerate more rapidly after mid life), in association with reduced antioxidant defence mechanisms, and mitochondrial dysfunction; data consistent with the predictions of the free-radical theory of aging. The current study, however, provides new insight into the potential mechanisms of aging involved in response to oxidative damage, particularly focusing on NAD^+^ metabolism and the roles of PARP and Sirt1 in the heart, lung, liver, and kidney (Fig. 10). Adequate NAD^+^ concentrations may therefore be an important longevity assurance factor.

**Figure 10:** Schematic representation for the association between oxidative stress, PARP-mediated and decline in NAD^+^ content, and NAD^+^ dependent functions with aging. Oxidative stress to DNA activates PARP leading to poly(ADP-ribosylation) of proteins in a reaction which consumes NAD^+^. Depletion of cellular NAD^+^ stores attenuates the activity of Sirt1 deacetylase leading to hyperacetylation of p53, and consequently tilting the balance to cell death via an apoptotic mechanism.

Therefore, we hypothesize that strategies targeted toward maintaining adequate NAD^+^ content during the aging process may prove a novel and potentially effective mechanism for retarding oxidative stress mediated cell degeneration, and age associated disorders.
